The article "The 22-Item Benefit Finding Scale: Validation and Application among Patients with Cervical Cancer in Ethnic Minority Areas of Southwestern China" was published in 2022. Journal: Contrast Media Mol Imaging.

# The 22-Item Benefit Finding Scale: Validation and Application among Patients with Cervical Cancer in Ethnic Minority Areas of Southwestern China

**DOI:** 10.1155/2022/8977011

**Published:** 2022-08-04

**Authors:** Zhouyuan Peng, Ke Liu, Yuting Zhang, Qingyu Hong, Liyuan Sun

**Affiliations:** Health Science Center, Shenzhen University, Shenzhen 518060, Guangdong, China

## Abstract

Recently, the Benefit Finding Scale (BFS) has been translated and culturally adapted for use in China. However, further validation of the instrument is required before it can be used in the management of patients with cervical cancer in China. In this study, we conducted the questionnaire survey and examined its properties. This methodological study was conducted at a tumor hospital located in southwestern China. Patients with cervical cancer who had been reexamined in the outpatient department of the hospital and hospitalized from June to August 2019 were selected. The item analysis, exploratory factor analysis (EFA), and reliability analysis were tested. The relationships between benefit finding and sociodemographic and disease-related variables were analyzed by ANOVA and regression models. A total of 247 patients were assessed (mean age: 48.0 ± 13.3 years). Educational level, self-perceived disease severity, and physical exercise were the predictors of benefit finding. The correlation coefficient between 22 items and their dimensions was the best. EFA analysis supported a five-factor model for structure validity. All Cronbach's alpha for the Chinese version of the BFS (BFS-C) was greater than 0.80. The results demonstrated the good reliability and validity of BFS-C. It appears to be a useful scale to assess experience of benefit finding among patients with cervical cancer in China.

## 1. Introduction

At present, cervical cancer remains one of the major public health problems in the world. It is the fourth highest incidence of malignancy in women worldwide, followed by breast cancer, colorectal cancer, and lung cancer [1]. According to research data, in 2018, there were approximately 570,000 new cases of cervical cancer worldwide, accounting for 3.15% of all malignant tumors. Among these cases, there were about 310,000 deaths, accounting for 3.26% of the total deaths of all malignant tumors [1, 2]. Cervical cancer is the sixth most common malignant tumor in Chinese women, and in China in 2020, there were 110,000 new cases of cervical cancer, resulting in 60,000 deaths [3]. In recent years, the incidence and death rates of cervical cancer in most countries throughout the world have shown a downward trend, while those in China still show an upward trend, especially in southwestern China [3, 4]. Therefore, cervical cancer poses a great threat to health and life of women in China.

With the development of positive psychology, studies have shown that although cancer is a life-threatening traumatic event, patients exhibit beneficial changes or personal growth experience, which helps cancer patients to accept cancer-related emotional and life changes, in turn promoting disease recovery [5]. At present, research on post-traumatic growth (PTG) [6] and benefit finding (BF) [7] is relatively extensive. Although the concepts of the two are similar, they are different in clinical practice. PTG refers to the positive psychological changes experienced by individuals after struggling with traumatic negative life events and situations and emphasizes the positive changes experienced after going through rumination and cognitive reconstruction [6]. Meanwhile, BF emphasizes the acquisition of benefits, which may occur after disease diagnosis [7, 8]. BF assesses the broader and less specific positive changes compared to PTG, and the adversity is not necessarily traumatic [9].

At present, most scales for evaluating BF have been developed in Western countries. There are many variations of BF, with relatively mature applications. As early as 2001, according to the cognitive adaptation theory, a single-dimensional Benefit Finding Scale (BFS), with a total of 17 items, was developed by Antoni et al. [10], in order to quantify the perceived benefits of breast cancer patients in diagnosis and treatment. It has been applied in the treatment of gynecological cancer [11], prostate cancer [12], and head and neck cancer [13] in many countries such as the US, Germany, and China. Later, it was revised by Tomich and Helgeson [14] in light of the positive contribution rate scale to evaluate the impact of early breast cancer on patients' positive lifestyle. There were 20 items in the final scale, which still consisted of a single dimension. In 2008, the relevant items of health behavior were added by Weaver et al. [15] based on the integration of all versions of the BFS so as to fully elucidate the positive changes made by cancer patients in numerous aspects, finally forming a BFS with six dimensions and 22 items. This scale is only recommended to be used among cancer patients because it is clearly disease-specific.

In recent years, although the research on BF in China is increasing [16–20], it remains in its infancy, and the scales used in the research have been introduced from other countries. In 2013, Antoni's original single dimension BFS [10] was translated into Chinese by Wang et al. [21], with the aim of measuring the BF level of breast cancer patients in China. It was then applied by Chinese scholars to the study of cervical cancer patients, but the reliability and validity of the scale were not verified. In 2014, the scale revised by Tomich et al. [14] was translated by Hu [22] into Chinese, forming a Chinese version of the BFS with 19 items. In 2015, in order to provide an evaluation tool suitable for Chinese cancer patients to measure BF, Liu et al. [23] performed cross-cultural adjustment on Weaver's scale [15], and the dimensions and items of the final scale were the same as those of the source scale.

Throughout the research on BF and its influencing factors, such as the patient's education level [24, 25], income [14–26], disease diagnosis time [27, 28], and cancer type [15–27], the opposite conclusions have been reached in many studies. These contradictory results may be due to the different BF evaluation scales used by researchers, and the results differ accordingly [29]. The same is true in China; the scale of BF used in mainland Chinese is different, and thus, the study results are inconsistent, making it difficult to conduct meta-analysis on the results of quantitative research.

Some scholars believe that Weaver's six-dimensional BFS is superior to the other scales [18] in evaluating the BF effect on cancer patients. However, it has only been introduced to mainland Chinese in recent years and has not been widely applied yet, and the validity of this scale among cancer patients remains to be verified. In addition, China's research on cervical cancer patients' BF is less mature than that of breast cancer patients. Cervical cancer patients who are plagued by China's traditional beliefs often have more serious psychological and behavioral problems than patients of other diseases due to the difficulty in bearing the responsibilities of childbearing and taking care of their families. Therefore, this group requires more attention from scholars, particularly those in ethnic minority areas, regarding whom the research is almost nonexistent. Consequently, this study, taking cervical cancer patients in ethnic minority areas as the research subjects, tests the psychometric characteristics of the Chinese version of the BFS (BFS-C) and analyzes the relationship between BF and sociodemographic and disease-related variables so as to provide relevant evidence for measuring BF of cervical cancer patients in China.

## 2. Materials and Methods

### 2.1. Sample and Recruitment

This methodological study was conducted at a tumor hospital located in southwestern China. Patients with cervical cancer who had been reexamined in the outpatient department of the hospital and hospitalized from June to August 2019 were selected. The inclusion criteria were as follows: ① age: 18–75; ② patients with cervical cancer diagnosed by pathology and treated with surgery and/or radiotherapy and chemotherapy, without significant disease progression at present; ③ no serious mental disorder or central nervous system disease. The exclusion criteria were as follows: ① patients with other cancers; ② those being treated with other psychotherapy and psychotropic drugs; ③ those participating or participated in other research studies.

This study took exploratory factor analysis (EFA) as a precondition to determine the sample size. A sample of at least 200–300 or a minimum of 10 participants for each item for EFA has been suggested to reduce the error rate [29, 30]. The current analysis only involved the psychometric characteristics of the BFS, the level of BF and its correlation with sociodemographic characteristics, and disease-related variables. This study took 10 times the total number of items as the sample size. Considering that there may have been up to 20% invalid questionnaires, the final sample size was 264. A total of 247 valid questionnaires were collected, for an effective recovery rate of 93.6%.

### 2.2. Measures

#### 2.2.1. Questionnaire on Sociodemographic and Clinical Manifestations

This customized questionnaire is mainly aimed at collecting basic information on patients. It included sociodemographic characteristic data (age, ethnic minority, occupation, education level, marital status, economic income, personality type, etc.) and disease-related data (self-perceived disease severity, daily exercise time, etc.).

#### 2.2.2. 22-Item Benefit Finding of Cancer Patient Scale-Chinese (22-Item BFS-C)

The reliability and validity of this scale were evaluated among breast cancer patients and early cancer patients, and good results were acquired. The scale consisted of six dimensions: acceptance (items 1–3), family relations (items 4–5), world outlook (items 6–9), personal growth (items 10–16), social relations (items 17–19), and healthy behavior (items 20–22). Each item was asked in the form of, “suffering from cancer (the experience from diagnosis to present).” The Likert 5-level scoring method was adopted with the score ranging from 1 to 5, respectively, indicating “completely absent,” “somewhat,” “moderate,” “considerable,” and “quite a lot.” The total score was the sum of the item scores, with a total score of 22–110 points. The higher the score, the stronger the sense of BF from the disease.

### 2.3. Data Collection

The subjects of this study were outpatients of gynecological tumor follow-up and inpatients hospitalized in the wards. Based on their medical records and mental state, their eligibility to participate in the study was determined. For those who were qualified to participate, the researchers first introduced the purpose, content, and methods of the study to them in order to obtain their understanding and support. After signing the informed consent form, the subjects took the survey in a quiet and undisturbed environment. If the patient was unsure about any of the questions, then the researchers would provide one-to-one interpretation. Each survey was completed in about 20 minutes, and the questionnaires were collected immediately afterward. The researchers were involved throughout the questionnaire survey process so as to ensure the authenticity of the data collected. The research data were then input by two people to ensure the accuracy of data entry and prevent data omission and deviation.

### 2.4. Data Analysis

#### 2.4.1. Sociological Characteristics of Subjects and Analysis of the Influencing Factors of BF

The data were sorted and preliminarily processed with Excel 2019 software and then analyzed with SPSS 26.0 statistical software. Pearson correlation, *t*-test, and one-way ANOVA were used to test the correlation between the BF level of patients with cervical cancer and sociodemographic and disease-related variables. Multiple linear regression analysis was used to explore the affecting factors of BF [31]. The statistical significance level was determined with *p* < 0.05.

#### 2.4.2. Reliability and Validity Test of the Scale

*(1) Item analysis*. The main goal of the study was to test the appropriateness or reliability of the scale or individual items [32]. Pearson correlation analysis and the critical ratio method were used for item analysis. The value of item-total correlation of >0.4 with statistical significance testing was considered to indicate a desirable discriminating power and the criteria-related validity. The extreme group (27% and 73% of the score of the BFS-C) comparison was performed using an independent-sample *t*-test.

*(2) Reliability analysis*. Reliability refers to the consistency or stability of the results obtained by using the test tool [32]. Cronbach's *α* coefficient was used to evaluate the internal consistency reliability of the scale [33], and Guttman's split-half coefficient was used to evaluate the split-half reliability. It is generally accepted that Cronbach's *α* coefficient ranging between 0.70 and 0.80 indicates quite good reliability and 0.80–0.90 very good reliability [32]. Since there was no repeated measurement in the scale, the test-retest reliability analysis could not be carried out.

*(3) Construct validity*. EFA was used to evaluate the construct validity of the scale. The purpose of using exploratory factors was to establish the construct validity of the scale or questionnaire [32]. Bartlett's spherical test was adopted to determine whether the scale was suitable for exploratory factor analysis. Kaiser–Meyer–Olkin (KMO) ≥ 0.8 and *p* < 0.05, indicating that there were common factors among the variables, which are suitable for factor analysis. The common factors were extracted by principal component analysis, and the selection conditions were eigenvalue >1.000 and factor loading ≥0.400 [34]. When the explained cumulative% variance was greater than 60%, this indicated that the retained factor was quite ideal [32] and that the scale had good construct validity.

### 2.5. Ethical Considerations

This study was approved by the Research Ethics Committee of the Health Science Centre, Shenzhen University. Each participant signed the informed consent form. It was necessary to keep the collected data completely confidential and not to leak any data so as to ensure the privacy and safety of the research subjects.

## 3. Results

### 3.1. Sample Characteristics

The average score of benefit finding of 247 subjects was 50.73 (SD = 10.15), with the average age among them being 48.0 years (SD = 13.30); 59 patients were of Han nationality (23.9%), and 188 were of ethnic minorities (including Hui, Bai, Naxi, and Yi); education level: 35 patients (14.2%) had primary school education or lower, 74 (30.0%) had junior middle school education, 92 (37.2%) had senior high school or technical secondary school education, and 46 (18.6%) held college degrees or above; 211 were married (85.4%), and 36 were single (unmarried, divorced, or widowed) (14.6%). 186 (75.3%) perceived their disease severity as moderate and severe, and 145 (58.7%) exercised at least 30 minutes a day, as shown in Table 1. The results of univariate analysis showed that the education level, marital status, self-perceived disease severity, and physical exercise bore statistically significant effects on the benefit finding of cancer patients (*p* < 0.05), as shown in Table 1. The multiple linear regression analysis results revealed that education, self-perceived disease severity, and physical exercise were the influencing factors of BF in patients with cervical cancer, as shown in Table 2.

### 3.2. Psychometric Properties of the 22-Item BFS-C

#### 3.2.1. Item Analysis

The scores of the scale were ranked from high to low. The first 27% with a score >57 was divided into the high score group, and the last 27% with a score <47 was divided into the low score group. The results of the *t*-test showed that there were significant differences in all items (*p* < 0.01). The critical ratio (CR value) of 22 items ranged between 9.626 and 18.657, as shown in Table 3. The correlation coefficient between each item and the total score of its corresponding dimensions was 0.713–0.927 (all *p* < 0.001), as shown in Table 3; the correlation coefficient among the six dimensions was 0.435–0.770 (all *p* < 0.001), and the correlation coefficient between each dimension and the total score was 0.726–0.932 (all *p* < 0.001), as shown in Table 4.

#### 3.2.2. Reliability Analysis

Overall Cronbach's *α* of this scale was 0.975. Cronbach's *α* of six dimensions, namely, acceptance, family relations, world outlook, personal growth, social relations, and healthy behavior, was 0.896, 0.822, 0.843, 0.965, 0.882, and 0.931, respectively. The split-half reliability of the scale was 0.940, and Guttman's split-half reliability coefficients of each dimension were 0.901, 0.822, 0.869, 0.948, 0.892, and 0.944, respectively.

#### 3.2.3. Construct Validity

The statistics of the scale were shown to be 0.956 by the KMO test, and the result of Bartlett's spherical test *χ*2 was 3,899.17 (*p* < 0.001). Since the KMO value was greater than 0.9, the data were suitable for factor analysis. A total of five factors were extracted by principal component analysis, and then, the factor division results were named according to their context and item content. Factor 1 was named “personal growth,” including seven items (*B*10–16); Factor 2 was “healthy behavior,” with three items (*B*20–22); Factor 3 was “family and social relations,” with seven items (*B*4–7, *B*17–19); Factor 4 was “acceptance,” with three items (*B*1–3); Factor 5 was “world outlook,” with two items (*B*8-9). The factor load matrix after rotation of the BFS-C is shown in Table 5.

## 4. Discussion

This study is the first trial using the 22-item BFS-C in China that was used to analyze the psychometric characteristics of BF in cervical cancer patients in ethnic minority areas. The verification results show that the scale had good validity and reliability.

The item analysis results showed that the correlation coefficient between 22 items and their dimensions was >0.4, while that between each dimension and the total score was also >0.4, thus indicating that the correlation coefficient was the best [35]. The CR values of 22 items were >9.0, indicating that the setting of each item was reasonable [32], and the test was reliable in the patients with cervical cancer. The reliability analysis results showed that overall Cronbach's *α* and the split-half coefficient of the scale were 0.975 and 0.940, respectively, while those of each dimension were >0.8. The higher the reliability coefficient, the lower the variation caused by the random error in the measurement process. Therefore, it was considered that the internal consistency of the scale was high [15].

In addition, in the “world outlook” dimension of the source scale, item 6 “tell me that everyone has a life goal” and item 7 “show me that everyone needs to be loved” were included in Factor 3. The reason for this may have been that different research subjects, cultural backgrounds, values, and customs will lead to varying perspectives; thus, there were some differences in common factors. As the subjects of this study were cervical cancer patients in southwestern China, there were many ethnicities in these areas (there are 55 ethnicities in China, among which more than 30 are distributed in southwestern China), thus constituting a multicultural complex [36]. Within this cultural context, people's understanding of life goals and being loved appears to have deviated from personal feelings, yet it is still closely related to family and social relations.

Next, the relationship between BF and sociodemographic and disease-related variables was also analyzed. The study results showed that the BF score of patients with cervical cancer was low; thus, it reminded us that there remains much room for improvement in this area. It was suggested that the medical staff identify patients with a low BF level as early as possible, guide them to view the disease from a positive perspective, and take corresponding intervention measures. In this study, education, self-perceived disease severity, and physical exercise were the influencing factors of BF in patients with cervical cancer. The results of previous studies performed in China [37] have also shown that the education level was a positive predictor of BF in patients with cervical cancer, since patients with a higher literacy level can view problems more rationally and thoroughly and actively seek appropriate self-regulation methods to improve their mental health [38]. In addition, self-perceived disease severity was positively correlated with BF. Previous studies have shown that the more severe the patient felt about their disease, the greater the possibility of cognitive and behavioral changes would be [39]. Exercise was an important factor affecting cancer patients [40] since moderate physical exercise, as a coping strategy, can release and alleviate psychological pressure so as to aid patients in becoming resilient to cancer [41].

## 5. Conclusions

The results of this study show that the 22-item BFS-C exhibits high reliability and validity and that it is an effective and reliable tool for measuring BF of cervical cancer patients in China. This study enriches the research results of psychological measurement characteristics of cancer patients, provides a unified measurement tool for scientific and effective analysis of BF of cervical cancer patients, and helps clinical medical staff understand the psychological status of patients in a timely manner so that they may carry out an effective and reasonable intervention.

### 5.1. Limitations

This study has several limitations. First, the participants were selected by convenient sampling of cervical cancer patients in southwestern China, and the limitations of which may affect the extrapolation of the results. Second, the limited sample size may have affected the accuracy of the results. Furthermore, we did not trace the differences in BF of patients in different periods. In the future, we will conduct longitudinal studies to explore the trajectory of BF change. In summary, it is advised to use a larger sample size and more diversified methods in various regions of China to further modify and improve the research results so as to further explore the applicability of the scale.

## Figures and Tables

**Table 1:** Demographic characteristics of the study sample (*N* = 247).

Categorical variables	*n*	%	*t*/*F*	*p*
Age			0.937	0.334
18–39	65	26.3		
40–59	113	45.7		
60 and above	69	27.9		

Ethnicity			0.004	0.952
Han	59	23.9		
Others	188	76.1		

Occupation			0.001	0.971
Worker	48	19.4		
Military or civil servant	27	10.9		
Professional technician	76	30.8		
Business or service industry	78	31.6		
Unemployed	43	17.4		
Farmer	84	34.0		
Others	59	23.9		

Level of education			0.512	0.045
Primary school	35	14.2		
Junior high school	74	30.0		
High school	92	37.2		
College degree or above	46	18.6		

Marital status			1.053	0.037
Married	211	85.4		
Single (unmarried, divorced, and widowed)	36	14.6		

Family per capita monthly income			0.389	0.533
5,000 yuan and below	106	42.9		
5,000–9,999 yuan	77	31.2		
10,000–14,999 yuan	30	12.1		
15,000–19,999 yuan	19	7.7		
20,000 yuan and above	15	6.1		

Form of medical security			2.497	0.115
Self-financed	43	17.4		
Provincial or municipal medical insurance	185	74.9		
Other insurance	19	7.7		

Are there any cancer patients in the family?			0.021	0.885
Yes	69	27.9		
No	178	72.1		

Self-assessment of current disease severity			4.076	0.018
0–3	61	24.7		
4–7	107	43.3		
8–10	79	32.0		

Exercise time per day			6.904	0.009
None	39	15.8		
Less than 30 minutes	63	25.5		
30 minutes to 1 hour	98	39.7		
More than 1 hour	47	19.0		

Therapeutic schedule			3.199	0.175
Operation	106	42.9		
Chemotherapy	97	39.3		
Radiotherapy	21	8.5		
Two or more	23	9.3		

**Table 2:** Multiple linear regression results of BF.

Independent variables	Unstandardized coefficients		Standardized coefficients	*t*	*p*
	B	Std. error			
Constant	70.192	7.204	46.289	9.743	<0.001

Self-assessment of current disease severity					
0–3	Ref				
4–7	3.198	1.437	3.199	2.065	0.028
8–10	2.860	2.512	2.860	2.738	0.007

Exercise time per day					
None	Ref				
Less than 30 minutes	0.186	2.157	0.180	0.053	0.957
30 minutes to 1 hour	1.025	2.092	1.025	0.490	0.625
More than 1 hour	4.583	2.691	4.584	2.211	0.036

Level of education					
Primary school	Ref				
Junior high school	0.189	1.936	0.119	0.074	0.793
High school	1.165	2.117	1.205	0.309	0.568
College degree or above	4.970	2.694	4.155	1.990	0.046

**Table 3:** Correlation analysis of each item of the BFS.

Item	*r*	CR
*B*1	0.848 ^*∗∗∗*^	12.408 ^*∗∗∗*^
*B*2	0.888 ^*∗∗∗*^	10.931 ^*∗∗∗*^
*B*3	0.872 ^*∗∗∗*^	14.146 ^*∗∗∗*^
*B*4	0.894 ^*∗∗∗*^	11.526 ^*∗∗∗*^
*B*5	0.899 ^*∗∗∗*^	10.499 ^*∗∗∗*^
*B*6	0.788 ^*∗∗∗*^	16.501 ^*∗∗∗*^
*B*7	0.713 ^*∗∗∗*^	12.622 ^*∗∗∗*^
*B*8	0.813 ^*∗∗∗*^	9.714 ^*∗∗∗*^
*B*9	0.750 ^*∗∗∗*^	9.626 ^*∗∗∗*^
*B*10	0.874 ^*∗∗∗*^	17.364 ^*∗∗∗*^
*B*11	0.886 ^*∗∗∗*^	16.925 ^*∗∗∗*^
*B*12	0.907 ^*∗∗∗*^	18.657 ^*∗∗∗*^
*B*13	0.887 ^*∗∗∗*^	16.778 ^*∗∗∗*^
*B*14	0.777 ^*∗∗∗*^	13.618 ^*∗∗∗*^
*B*15	0.879 ^*∗∗∗*^	14.554 ^*∗∗∗*^
*B*16	0.856 ^*∗∗∗*^	18.663 ^*∗∗∗*^
*B*17	0.882 ^*∗∗∗*^	14.357 ^*∗∗∗*^
*B*18	0.879 ^*∗∗∗*^	14.372 ^*∗∗∗*^
*B*19	0.868 ^*∗∗∗*^	14.948 ^*∗∗∗*^
*B*20	0.901 ^*∗∗∗*^	12.847 ^*∗∗∗*^
*B*21	0.909 ^*∗∗∗*^	12.270 ^*∗∗∗*^
*B*22	0.927 ^*∗∗∗*^	13.475 ^*∗∗∗*^

^*∗∗∗*^: *p* < 0.001; *B*1‒*B*22 : benefit finding items 1 to 22.

**Table 4:** Correlation analysis of each dimension of the BFS (*r* value).

Dimensions	Acceptance	Family relations	World outlook	Personal growth	Social relations	Healthy behavior	BFS scores
Acceptance	1						
Family relations	0.617 ^*∗∗∗*^	1					
World outlook	0.655 ^*∗∗∗*^	0.701 ^*∗∗∗*^	1				
Personal growth	0.662 ^*∗∗∗*^	0.556 ^*∗∗∗*^	0.701 ^*∗∗∗*^	1			
Social relations	0.615 ^*∗∗∗*^	0.590 ^*∗∗∗*^	0.653 ^*∗∗∗*^	0.770 ^*∗∗∗*^	1		
Healthy behavior	0.560 ^*∗∗∗*^	0.435 ^*∗∗∗*^	0.520 ^*∗∗∗*^	0.727 ^*∗∗∗*^	0.720 ^*∗∗∗*^	1	
BFS scores	0.804 ^*∗∗∗*^	0.726 ^*∗∗∗*^	0.842 ^*∗∗∗*^	0.932 ^*∗∗∗*^	0.861 ^*∗∗∗*^	0.794 ^*∗∗∗*^	1

^*∗∗∗*^: *p* < 0.001.

**Table 5:** Five factors extracted from the factor analysis using the matrix rotation.

Items in each factor	Factor 1	Factor 2	Factor 3	Factor 4	Factor 5
Personal growth					
*B*11	0.753				
*B*12	0.721				
*B*10	0.714				
*B*15	0.704				
*B*13	0.698				
*B*14	0.627				
*B*16	0.597				

Healthy behavior					
*B*21		0.806			
*B*22		0.796			
*B*20		0.764			

Family and social relations					
*B*4			0.749		
*B*5			0.729		
*B*7			0.719		
*B*18			0.591		
*B*17			0.546		
*B*19			0.541		
*B*6			0.523		

Acceptance					
*B*2				0.757	
*B*1				0.699	
*B*3				0.642	

World outlook					
*B*9					0.843
*B*8					0.748

Eigenvalue	10.12	3.44	2.20	1.17	1.16
% Variance explained	46.01%	15.63%	10.01%	5.32%	5.29%
Cumulative% variance explained	46.01%	61.64%	71.65%	76.97%	82.26%

## Data Availability

The data presented in this study are available from the corresponding author on request.
